The article "Early growth stages salinity stress tolerance in CM72 x Gairdner doubled haploid barley population" was published in 2017. Journal: PLoS One.

# Early growth stages salinity stress tolerance in CM72 x Gairdner doubled haploid barley population

**DOI:** 10.1371/journal.pone.0179715

**Published:** 2017-06-22

**Authors:** Tefera Tolera Angessa, Xiao-Qi Zhang, Gaofeng Zhou, Sue Broughton, Wenying Zhang, Chengdao Li

**Affiliations:** 1 Western Barley Genetics Alliance, School of Veterinary and Life Sciences (VLS), Murdoch University, Murdoch, WA, Australia; 2 Grains Industry, Department of Agriculture and Food WA, South Perth, WA, Australia; 3 Hubei Collaborative Innovation Centre for Grain Industry/College of Agriculture, Yangtze University, Jingzhou, Hubei, China; Zhejiang University, CHINA

## Abstract

A doubled haploid (DH) population of barley *(Hordeum vulgare* L.) generated from salinity tolerant genotype CM72 and salinity sensitive variety Gairdner was studied for salinity stress tolerance at germination, seedling emergence and first leaf full expansion growth stages. Germination study was conducted with deionized water, 150 mM and 300 mM NaCl treatments. Seedling stage salinity tolerance was conducted with three treatments: control, 150 mM NaCl added at seedling emergence and first leaf full expansion growth stages. Results from this study revealed transgressive phenotypic segregations for germination percentage and biomass at seedling stage. Twelve QTL were identified on chromosomes 2H–6H each explaining 10–25% of the phenotypic variations. A QTL located at 176.5 cM on chromosome 3H was linked with fresh weight per plant and dry weight per plant in salinity stress induced at first leaf full expansion growth stage, and dry weight per plant in salinity stress induced at seedling emergence. A stable QTL for germination at both 150 and 300 mM salinity stress was mapped on chromosome 2H but distantly located from a QTL linked with seedling stage salinity stress tolerance. QTL, associated markers and genotypes identified in this study play important roles in developing salinity stress tolerant barley varieties.

## Introduction

Soil salinity, a combination of sodic and saline soils, is one of the most important environmental factors affecting 10% to 20% of the world soil [1–3]. Salinity causes osmotic stress by decreasing availability of water to plant roots and plant water uptake. Excessive salts taken up by the plants can accumulate to toxic levels in certain tissues reducing growth and causing premature death of old leaves that reduces supply of assimilates to the growing regions [4,5].

Salinity reduces germination, growth, survival, development, yield and grain quality in barely despite the fact that it has been widely acknowledged as a crop that tolerates to salinity [2,4–9]. Salinity tolerance in barley varies from genotype to genotype [1,2,5–7,10,11]. Genotypic variation in salinity stress tolerance is due to genetic factors that are quantitative in nature [1,2,4,5,8,9,12]. Polygenic segregations for salinity tolerance in F2 –F4 generations has been reported for crosses made between salt tolerant genotypes Kumoi (OUJ417) and Jeomchon (OUK666) with a sensitive genotype Ethiopia 633 (OUE211) [1]. Thirty QTL were identified explaining 3–30% phenotypic variation of 10 traits that included yield, yield component and physiological traits at late stage in the CM72 x Gairdner doubled haploid population [2]. When genetic factors linked with salinity stress tolerance at different growth stages were compared, highly heritable QTL conferring salinity tolerance at germination stage were different from those QTL conferring salinity tolerance at seedling stage [1,2,5,8,9,12].

The article "Early growth stages salinity stress tolerance in CM72 x Gairdner doubled haploid barley population" was published in 2017. Journal: PLoS One.

Seed germination and seedling establishment are very good indicators of potential grain yield to be harvested at late stage. Seed germination is an important and vulnerable stage in the life cycle of terrestrial angiosperms and determines seedling establishment and plant growth [3]. Environmental factors such as salinity reduce seed germination, seedling establishment and performance. Previous studies reported that salinity impairs seed germination, seedling emergence, leaf elongation and biomass accumulation at early growth stages [3,4,9,13,14]. Salinity affects leaf growth in the short and long term [14]. Improving salinity stress tolerance at germination stage increases plant population establishment, while seedling stage salinity stress tolerance enhance accumulation of biomass that lays a basis of high grain yield. This is especially important in the Mediterranean environment characterized with dry and hot summer [15], which results in increasing salinity before seeding in the autumn. This improvement is best achieved by the identification of genetic factors linked with salinity stress tolerance at germination and seedling stages.

Phenotypic variation explained by genetic factors in barley under salinity stress conditions is the basis for developing improved varieties for cultivation in regions prone to salinity stress. Identification of the loci linked with salinity stress tolerance will provide an efficient approach to breed salinity tolerance through marker-assisted selection. In line with this view, this study was conducted on a barley doubled haploid population generated from the cross of salinity stress tolerant genotype CM72 and salinity stress sensitive Australian barley variety Gairdner to assess loss of germination due to salinity stress, to evaluate biomass yield loss due to salinity stress induced at seedling growth stages, and to map QTL linked with salinity stress tolerance at germination and seedling growth stages.

The article "Early growth stages salinity stress tolerance in CM72 x Gairdner doubled haploid barley population" was published in 2017. Journal: PLoS One.

## Materials and methods

### Genotypes

In total 104 barley genotypes, which included 102 doubled haploid (DH) lines produced from parental genotypes CM72 and Gairdner, were tested for salinity stress tolerance. CM72 is a salinity stress tolerant genotype with a pedigree of California Mariout*4/CI1179 (Algerian)//2*California Mariout/Club Mariout/3/CM67. Gairdner is an Australian barley variety with a pedigree of Tas83-587/ Onslow.

### Study stages

The effect of salinity stress was assessed at germination, at seedling emergence, and at first leaf full expansion growth stages. In addition, all the genotypes were grown at South Perth field plots of the Department of Food and Agriculture WA, Australia and plant height of each individual line was recorded at maturity.

### Germination test

Three sets of 100 seeds per genotype were spread on a layer of two filter papers Whatman No1 placed in a 90mm petri dish. Each of the three petri dishes with seeds of a DH line was assigned to three different treatments namely (1) control treatment in 4 ml deionized water without NaCl, (2) 4 ml 150mM NaCl treatment, and (3) 4 ml 300mM NaCl treatment. Each petri dish was labeled and covered with its lid. A group of 10 petri dishes were bundled together with cling wrap, and placed in an incubator at 20° C temperature with no light. Seeds with any sign of germination were counted after 72 hours of incubation.

### Biomass yield at seedling emergence and first leaf growth stages

An automated hydroponic system located at Shenton Park Research Station of University of Western Australia was used to assess the effect of salinity stress on total biomass yield at seedling emergence and first leaf full expansion growth stages. Treatments were assigned to three nutrient solution tanks (NST), each with a maximum 300 liter volume capacity. Each NST was connected to two concrete tanks filled with river sand (RST) and used as replications. The concrete tanks were cylindrical in shape with six cm thickness, 90 cm height, 1.08 m internal diameter, and 3.75 m external circumference.

The automated hydroponic system was setup to pump the solution for one minute every hour. The system pumped the water/ solution through an irrigation hose connected to specially designed, branched and perforated fittings made from PVC for uniform supply of water/ solution to all genotypes planted in the sand tanks. Excess water/ solution percolated through the sand were discharged back to the NST through irrigation hoses fitted with filters at the bottom of the RSTs. The system was designed to simulate the salinity stress environment in the field.

The article "Early growth stages salinity stress tolerance in CM72 x Gairdner doubled haploid barley population" was published in 2017. Journal: PLoS One.

### Nutrients

Trials to assess the effect of salinity stress on seedling biomass yield were established with 12 seeds per genotype. The seeds were germinated with tap water. Macro-nutrients, bivalents, micro-nutrients, and iron-EDTA (ethylene diamine tetra-acetic acid) were added to all three NSTs six days after planting. About 2.5 liters of macro- nutrients was added to all NST. The macro-nutrient solution was prepared from 156 g MW (Molecular Weight) sodium dihydrogen orthophosphate, 101.1 g MW potassium nitrate and 142.1 g MW Sodium sulfate. About 2.5 liters of bivalents prepared from 156.5 g MW calcium chloride, 203.3 g MW magnesium chloride was added to the NSTs. About 0.83 liters of micro-nutrients was added to the NST. The micro-nutrients solution was prepared from 61.84 g MW borate, 197.9 g MW Manganese chloride, 249.7 g MW Cupric sulfate, 287.6 g MW Zinc sulfate, 1236 g MW Ammonium molybdate. About 0.83 liters of iron-EDTA (ethylene diamine tetra-acetic acid) prepared from 367.1 g MW ferric monosodium was added to all three NSTs.

### Treatments

The control treatment received no NaCl, while treatment number 1 and 2 received 150 mM NaCl stress but at two different stages. Salinity stress in treatment number 1 was induced 6 days after planting when about 50% of the seedlings emerged; while treatment number 2 was induced at 13 days after planting when about 50% of the genotypes had their first leaf fully expanded. The NSTs were topped up with tap water and proportional amount of nutrient solution and NaCl as appropriate on three different occasions.

### Harvesting

The first replication of each of the three treatments was harvested at 30–31 days after seeding and total plant fresh weight recorded. The second replication of each of the three treatments was harvested at 34 days after seeding. Plants that were harvested and their fresh weight recorded on both occasions were oven-dried at 60°C for 72 hours and their dry weight recorded.

### Phenotypic salinity tolerance measurement

Germinated seeds were expressed in percentage and subjected to statistical data analysis. Furthermore each genotype’s germination percentage and biomass yield was expressed as a ratio of that recorded in control treatment. Genotypes with biomass yield percentage less than 100% had their yield reduced due to salinity stress. Thus, they were salinity stress susceptible lines. This was in contrast to genotypes with biomass yield percentage higher than 100%, which were salinity stress tolerant.

### Data analysis

Individual genotype’s germination percentage and mean of biomass yield from two replications recorded from two RST were used for statistical analysis. The analysis of variance was performed by PLABSTAT [16]. A computer program SPSS was used for Spearman’s rank correlation coefficient analysis and plotting the graphs [17].

The article "Early growth stages salinity stress tolerance in CM72 x Gairdner doubled haploid barley population" was published in 2017. Journal: PLoS One.

### QTL mapping

Three hundred and fifteen Diversity Array Technology (DArT) markers and 84 Simple Sequence Repeat (SSR) markers and phenotypic data were subjected to MapQTL5.0 [18] to identify Quantitative Traits Loci/ locus (QTL) linked with plant height at maturity, germination percentage in salinity stress, biomass yield at seedling emergence and first leaf full expansion growth stages. A LOD score threshold of 2.7 at *P < 0*.*05* was used to declare a QTL linked with germination percentage or seedling stages biomass yield in the CM72 x Gairdner DH population.

## Results

The CM72 x Gairdner doubled haploid population exhibited substantial transgressive phenotypic variations in response to salinity stress for germination percentage, and biomass yield at seedling emergence and first leaf full expansion growth stages. The analysis of variance of the data on germination percentage and biomass yield revealed that a very highly significant differences existed between the genotypes and between the treatments (Table 1). Treatment effect was larger than the effect due to genotypes.

**Table 1:** Analysis of variance (ANOVA) table performed on germination percentage (Grm), fresh weight per plant (FWt), dry weight per plant (DWt).

Trait	Source	DF	SS	MS	Variance component	F	s.e.	LSD5	Broad sense Heritability
Grm	Genotype (G)	99	35178.1	355.3	71.8	2.54**	6.83	19.06	60.6
	Treatment (T)	2	165094.2	82547.1	824.1	589.36**	1.18	3.3	
	GxT	198	27732.5	140.1	140.1				
	Total	299	228004.8						
FWt	Genotype (G)	98	51.91	0.53	0.14	5.33**	0.18	0.51	81.3
	Treatment (T)	2	18.69	9.35	0.09	94.15**	0.03	0.09	
	GxT	195	19.36	0.10	0.10				
	Total	295	89.96						
DWt	Genotype (G)	98	1.17	0.01	0.0006	6.82**	0.02	0.07	85.3
	Treatment (T)	2	0.16	0.08	0.0006	44.82**	0.00	0.01	
	GxT	195	0.34	0.00	0.0002				
	Total	295	1.67						

**Significant at 1% probability level.

### Germination test

The overall average germination percentage recorded in deionized water, 150 mM NaCl and 300 mM NaCl treatments were 96%, 82%, and 41%, respectively. The 300 mM NaCl treatment caused an overall 59% average germination percentage loss compared to 18% in the 150 mM NaCl treatment.

Individual genotype’s salinity tolerance was measured by the ratio of germination percentage in salinity stress treatments to germination percentage in deionized water treatment. Salinity stress tolerance of CM72 was demonstrated by 94.9% germination percentage ratio in 150 mM NaCl treatment compared to salinity stress susceptible parental genotype Gairdner that exhibited a ratio of 72.2% (Fig 1A). The severity of the 300 mM NaCl treatment on seed germination was reflected by highly reduced germination ratio of 70.7% in CM72 and 24.7% in Gairdner (Fig 1B).

The article "Early growth stages salinity stress tolerance in CM72 x Gairdner doubled haploid barley population" was published in 2017. Journal: PLoS One.

**Fig 1:** Germination stage salinity stress effect on barley CM72 x Gairdner doubled haploid population. Ratio of germination percentage (A) in 150 mM NaCl treatment to deionized water treatment, and (B) in 300 mM NaCl treatment to deionized water treatment.

The DH lines exhibited transgressive segregation of germination percentage both in the 150 mM and 300 mM NaCl treatments (Fig 1A and Fig 1B). Compared with parental genotype, seven lines scored better germination percentage ratio than salinity stress tolerant parental genotype CM72 in both 150mM and 300 mM NaCl treatments. This observation was in contrast to 10 lines which scored lower germination percentage ratio than that of salinity susceptible parental genotype Gairdner.

### Seedling test

Assessment of biomass yield in the CM72 x Gairdner DH population for response to salinity stress revealed that the population varied substantially in fresh weight per plant (Fig 2A and 2B) and dry weight per plant (Fig 2C and 2D).

**Fig 2:** Seedling stages salinity stress effect on barley CM72 x Gairdner doubled haploid population. Fresh weight per plant (A & B); dry weight per plant (C & D)ratio in salinity stress treatments to that in control treatment and expressed in percentage.

#### Salinity tolerance at seedling emergence stage

In the treatment where salinity stress was induced with 150 mM NaCl at seedling emergence growth stage, salinity stress tolerant genotype CM72 produced a fresh weight ratio of 78%, which was higher than 62.7% observed in salinity sensitive genotype Gairdner (Fig 2A). The dry weight biomass observed in the two parental genotypes contrasting in their salinity stress was 80.2% in CM72 and 73.9% in Gairdner (Fig 2C). Across the whole population, fresh biomass yield ratio in salinity stress at seedling emergence growth stage ranged from15–148%, dry biomass yield ranged from 22–160%. Twenty nine DH lines yielded higher fresh biomass than salinity stress tolerant parental genotype CM72 in contrary to 46 DH lines that yielded lower fresh biomass than salinity stress sensitive parental genotype Gairdner.

#### Salinity tolerance at first leaf full expansion growth stage

The superiority of CM72 salinity stress tolerance was apparent for fresh weight per plant (Fig 2B) and dry weight per plant (Fig 2D) when salinity stress was induced at first leaf full expansion growth stage. CM72’s 125.3% fresh weight ratio was higher than 71.4% ratio observed in Gairdner. A dry weight ratio of 136.9% in CM72 was also higher than 92.2%ratio recorded with Gairdner.

The article "Early growth stages salinity stress tolerance in CM72 x Gairdner doubled haploid barley population" was published in 2017. Journal: PLoS One.

Comparing salinity stress effect at early growth stages, reduction in biomass yield in salinity stress susceptible lines was as high as 85.1%, 64.7% fresh weight per plant; 77.9%, 53.4% dry weight per plant respectively in salinity stress induced at seedling emergence and first leaf full expansion growth stages. This was in contrast to salinity stress tolerant lines that yielded as as 47.8%, 49.5% fresh weight per plant; 59.7%, 105.7% dry weight per plant observed respectively in salinity stress treatments induced at seedling emergence and first leaf full expansion growth stages. Despite large number of lines were susceptible to salinity stress, a few lines were observed to promisingly stress tolerant types (Fig 2). In total 10 lines in salinity stress treatment induced at seedling emergence stage and 20 lines in salinity stress treatment induced at first leaf expansion stage yielded a fresh biomass ratio of higher than 100%. Among these lines, eight lines yielded fresh biomass ratio of higher than 100% in salinity stress treatments at seedling emergence and first leaf full expansion growth stages.

### Association between traits

A very highly significant genotypes Spearman’s rank correlation coefficient (r = 0.98^**^) was observed between fresh weight per plant and dry weight per plant in all the three tratments (Table 2).

**Table 2:** Spearman’s rank correlation coefficient between CM72 X Gairdner doubled haploid barely lines evaluated for salinity tolerance.

Traits		Germination percentage (%).			Fresh weight Per plant (g).			Dry weight per plant (g).		
	Treatments	DI Water	150mM NaCl	300 mM NaCl	Ctl	Tr1	Tr2	Ctl	Tr1	Tr2
Germination percentage (%).	DI Water	1.00								
	150NaCl	0.40**	1.00							
	300NaCl	0.13	0.56**	1.00						
Fresh weight Per plant (g).	Ctl	0.30**	0.27**	0.23*	1.00					
	Tr1	0.06	-0.03	0.08	0.49**	1.00				
	Tr2	-0.04	-0.04	0.01	0.71**	0.72**	1.00			
Dry weight per plant (g).	Ctl	0.29**	0.24*	0.21*	0.98**	0.47**	0.73**	1.00		
	Tr1	0.09	-0.04	0.10	0.48**	0.98**	0.74**	0.48**	1.00	
	Tr2	-0.01	-0.02	0.05	0.69**	0.67**	0.98**	0.73**	0.72**	1.00

DI–deionized water for germination percentage evaluation; Ctl–control treatment with no salinity stress; Tr1 –seedling emergence stage and Tr2 –first leaf full expansion growth stage salinity stress induced with 150 mM NaCl.

A very high correlation observed between fresh weight per plant and dry weight per plant and also a high broad-sense heritability of these two traits (Table 1) strongly indicate that selection for one of the traits is indicative of the other trait. Because assessment for fresh weight requires fewer resources such as time and an oven to dry out the fresh biomass, this trait has practical applicability in screening barley genotypes for salinity stress at early growth stages. Alternatively, this trait can be scored visually in the field for biomass yield and superior genotypes identified in the field easily.

The article "Early growth stages salinity stress tolerance in CM72 x Gairdner doubled haploid barley population" was published in 2017. Journal: PLoS One.

In general, the CM72 x Gairdner DH lines exhibited phenotypic transgressive segregations compared with their parental genotypes in germination percentage (Fig 1), fresh weight per plant and dry weight per plant (Fig 2). These substantial phenotypic variations for salinity stress tolerance in this DH population were the basis to identify QTL associated with salinity stress tolerance at various growth stages.

### QTL linked with salinity stress tolerance at germination and seedling stages

QTL mapping was conducted with MapQTL5.0 software. Putative QTL associated with a trait was delineated at a minimum LOD score of 2.7. This assessment identified 12 QTL associated with germination percentage in salinity stress treatments, biomass yield at seedling growth stages, or plant height in salinity stress free field environments (Fig 3, Table 3).

**Fig 3:** Salinity stress tolerance linked QTL identified in CM72 x Gairdner doubled haploid population. QTL linked with germination percentage in NaCl treatments of 150 mM (GP_150_), 300 mM (GP_300a_,GP_300b_); fresh weight per plant in control treatment (FW_ct_), fresh weight per plant in 150 mM NaCl treatments at seedling emergence (FW_em1_, FW_em2_, FW_em3_), and fresh weight per plant at first leaf expansion (FW_ex1_, FW_ex2_); dry weight per plant in control treatment (DW_ct_), dry weight per plant in 150 mM NaCl treatments at seedling emergence (DW_em1_, DW_em2_), and dry weight per plant at first leaf expansion (DW_ex1_, DW_ex2_)in a hydroponic study; and QTL linked with plant height at maturity (Ht_1_, Ht_2_).

**Table 3:** Quantitative Traits Loci (QTL) linked with salinity stress tolerance at seed germination, seedling emergence and first leaf full expansion growth stages, and their chromosomal locations, percentage of phenotypic variations explained by a QTL, LOD scores, and parental salinity tolerance source (CM72 or Gairdner).

Method	Treatment	Trait	QTL	Chromosome	QTL ID	Marker	Position	LOD	%age explained	Tolerance source
**Germination**	150 mM NaCl	Germination percentage	1	2H	GP150	bPb-3858	160.2	4.10	21.8	CM72
	300 mM NaCl	ʺ	1	2H	GP300a	bPb-1103	156.6	4.10	16.1	CM72
	300 mM NaCl	ʺ	2	5H	GP300b	bPb-8775	78.4	2.70	10.0	Gairdner
**Hydroponic evaluation**	Control	Fresh weight/ plant (g)	1	2H	FWct	Bmag0125	80.0	3.08	14.1	Gairdner
		Dry weight/ plant (g)	1	3H	DWct	bPb-1579	159.8	2.92	13.5	CM72
	150 mM at 50% seedling emergence	Fresh weight/ plant (g)	1	3H	FWem1	bPb-3634	192.8	3.99	14.2	CM72
		ʺ	2	4H	FWem3	HVM67	236.2	3.20	11.7	Gairdner
		ʺ	3	6H	FWem2	Bmag0870	52.6	3.61	12.3	CM72
		Dry weight/ plant (g)	1	3H	DWem1	bPb-6504	176.5	4.03	18.0	CM72
		ʺ	2	6H	DWem2	Bmac0298	58.1	3.80	15.1	CM72
	150 mM at 50% full 1st leaf expansion	Fresh weight/ plant (g)	1	2H	FWex2	Bmag0125	80.0	3.59	14.1	Gairdner
		ʺ	2	3H	FWex1	bPb-6504	176.5	5.26	21.6	CM72
		Dry weight/ plant (g)	1	2H	DWex2	Bmag0125	80.0	2.93	11.1	Gairdner
		ʺ	2	3H	DWex1	bPb-6504	176.5	6.17	25.2	CM72
**Field**	Field environment	Plant height (cm)	1	2H	Ht1	bPb-2603	118.6	3.14	12.3	CM72
		ʺ	2	3H	Ht2	bPb-1961	161.1	5.50	22.7	CM72

The article "Early growth stages salinity stress tolerance in CM72 x Gairdner doubled haploid barley population" was published in 2017. Journal: PLoS One.

#### QTL at germination stage

Two closely located QTL on chromosome 2H in the region of 156–160.2 cM were linked with germination percentage in 150 mM and 300 mM NaCl stress treatments (Fig 3, Table 3). These two QTL linked with markers bPb-3858 and bPb-1103 were contributed by CM72, and explained, respectively, ~22% and 16% of the observed germination percentage variations in the DH population due to 150 NaCl mM, and 300 mM NaCl treatments. Salinity stress susceptible Gairdner contributed a QTL on chromosome 5H at 78.4 cM linked with germination percentage in the 300 mM NaCl treatment. This QTL explained 10% of the observed variations in germination percentage.

#### Seedling stage linked QTL

Over all 11 QTL were identified to be linked with seedling stage biomass yield in control or salinity stress treatments induced at seedling emergence or first leaf full expansion growth stage (Fig 3, Table 3).

#### QTL in control treatment

Two QTL were identified in the control treatment on chromosomes 2H (FWct) and 3H (DWct) controlling fresh weight per plant and dry weight per plant, respectively (Fig 3, Table 3). The QTL on chromosome 3H located at a distance of 159.8 cM was contributed by CM72. It explained 13.5% of the observed phenotypic variation in dry weight per plant. The QTL on chromosome 2H was contributed by Gairdner and explained 14.1% fresh weight per plant phenotypic variations.

#### QTL in salinity stress treatment at seedling emergence stage

Three QTL associated with fresh weight per plant were detected on chromosome 3H at a distance of 192.8 cM, on chromosome 4H at a distance of 236.2 cM, and on chromosome 6H at a distance of 52.6 cM in salinity stress treatment induced at seedling emergence growth stage (Fig 3, Table 3). The QTL on chromosomes 3H identified by a marker bPb-3634 and the QTL on chromosome 6H identified by a marker Bmag0870 were both contributed by CM72 and explained, respectively, 14% and 12% of the observed phenotypic variations of fresh weight per plant. The CM72 contributed QTL on chromosomes 3H and 6H linked with fresh weight per plant were located respectively at a distance of 16.6 cM and 5.5 cM from the QTL linked with dry weight per plant in the salinity stress induced at seedling emergence growth stage (Fig 3, Table 3).

The article "Early growth stages salinity stress tolerance in CM72 x Gairdner doubled haploid barley population" was published in 2017. Journal: PLoS One.

#### QTL in salinity stress treatment at first leaf full expansion growth stage

The same QTL was identified to control fresh weight per plant and dry weight per plant in the salinity stress environment induced at first leaf full expansion growth stage (Fig 3, Table 3). Gairdner contributed QTL on chromosome 2H, which explained 14% fresh weight per plant and 11% dry weight per plant of the observed phenotypic variations. The highest phenotypic variations of 22% fresh weight per plant and 25% dry weight per plant of the DH population were explained by the CM72 contributed QTL on chromosome 3H.

### Plant height linked QTL

The CM72 x Gairdner doubled haploid population varied considerably for plant height at maturity. It varied from as short as 25 cm to as tall as 80 cm plant height. Such considerable variations in plant height in this population prompted the need to assess if there is genetic factor linked with plant height and if plant height and salinity stress tolerance linked QTL were collocated.

QTL mapping detected two QTL linked with plant height at maturity (Fig 3, Table 3). Both QTL were contributed by CM72. The QTL on chromosome 2H explained 12% of the observed phenotypic variation in plant height, which was almost half of ~23% phenotypic variation explained by the QTL on chromosome 3H.

Considering the position of the QTL linked with plant height at maturity and seedling stage biomass yield, the plant height linked QTL on chromosome 3H was located at a distance of 15.4 cM away from QTL linked with dry weight per plant in seedling emergence and first leaf expansion stress treatments, and fresh weight per plant in first leaf expansion stress treatment. This plant height QTL was located distantly at 31.7 cM away from a QTL associated with dry weight per plant in stress treatment induced at seedling emergence. However, it was closely located at 1.3 cM distance from dry weight per plant linked QTL in salinity stress free control treatment. The QTL on chromosome 2H linked with plant height at maturity and biomass yield at seedling stage in salinity stress free control treatment and 150 mM NaCl treatment at first leaf expansion growth stage were distantly located at 38.6 cM from each other.

## Discussion

The CM72 x Gairdner doubled haploid (DH) population exhibited transgressive phenotypic variations for traits assessed in salinity stress treatments induced at germination (Fig 1), seedling emergence and first leaf full expansion growth stages (Fig 2). Analysis of variance of data on germination percentage and seedling biomass yield revealed very highly significant variations between the genotypes and the treatments. Twelve QTL are identified explaining 10–25% of the phenotypic variations in the population for all traits assessed in this study.

The article "Early growth stages salinity stress tolerance in CM72 x Gairdner doubled haploid barley population" was published in 2017. Journal: PLoS One.

### Phenotypic traits

The overall germination percentage recorded in the CM72 x Gairdner DH population is 96%, 82%, 41%, respectively, in deionized water, 150 mM NaCl, and 300 mM NaCl treatments. A loss of 59% germination percentage in 300 mM NaCl is very severe compared with 18% loss in 150 mM NaCl treatment. This result reflects the fact that the severity in loss of germination due to salinity increases as the salt concentration increases. Results from this study corroborates previous reports that salinity stress impedes barley seed germination, growth and development processes [4,9,13].

Salinity stress not only inhibits germination but also decreases leaf elongation, seedling emergence and biomass accumulation at early growth stages. It was reported that leaf elongation decreased close to zero within seconds following the addition of NaCl [14]. They reported that elongation velocity recovered rather abruptly to about 46% of the pre-stress level between 20 and 30 minutes after exposure. The recovery reached about 70% after five days compared to leaf elongation in non-stressed plants. A biomass reduction as high as 68% in Clipper and 64% in Arivat was reported after exposing these salinity sensitive barley genotypes to 175 or 250 mM NaCl for 30 days [4]. In barley genotypes that were considered as salinity stress tolerant types, the biomass reduction was 38% in ELB 14, 50% in Californian Mariout and 56% in Beecher [4]. A study with 6172 barley varieties from diverse origin and 368 isogenic barley lines for salinity stress tolerance revealed that varieties from China and Korea are more tolerant than barley varieties from Turkey and Japan [5]. It was claimed that six-rowed, naked and non-uzu types are more salinity tolerant than their phenotypic counterparts. Our study demonstrated that salinity stress tolerance in the CM72 x Gairdner doubled haploid (DH) population ranged from very sensitive level to highly tolerant level at germination and seedling growth stages. Salinity stress sensitive lines had a reduction of 85% and 65% fresh weight per plant in 150 mM NaCl treatments induced, respectively, at seedling emergence and first leaf expansion seedling growth stages. Such considerable loss in biomass yield in the sensitive lines is in contrary to salinity stress tolerant DH lines of the CM72 x Gairdner population that yielded rather higher fresh weight per plant of ~48% and ~50% in salinity stress induced, respectively, at seedling emergence and first leaf full expansion growth stages. Variation in salinity stress tolerance observed in the current study is partially attributed to genetic factors that can be explained by Quantitative Traits Loci (QTL).

The article "Early growth stages salinity stress tolerance in CM72 x Gairdner doubled haploid barley population" was published in 2017. Journal: PLoS One.

### Salinity stress tolerance linked Quantitative Traits Loci (QTL)

Overall 12 QTL were identified to be linked with salinity stress at germination stage, seedling emergence and first leaf full expansion growth stages. These QTL were located on five chromosomes (2H – 6H) of barley and explained 10–25% of the observed phenotypic variations. A study that used the same DH population included in this study mapped a total of 30 QTL that accounted for 3–30% late stage phenotypic variations of seven agronomic and three physiological traits on all 7 chromosomes [2].

Among 12 QTL identified in this study, three QTL are linked with salinity stress tolerance at germination (Fig 3, Table 3). Two of germination stage salinity stress tolerance QTL identified in this study are located on chromosome 2H close to the sodium concentration linked QTL reported previously [2]. Because the majority of the two QTL regions on chromosome 2H overlap and the genetic distance between the two QTL peaks is 3.6 cM, it is likely that these are the same QTL controlling germination percentage in varying level of salinity stress treatments. The third QTL linked with germination stage tolerance is mapped on chromosome 5H. This QTL is slightly distant from potassium concentration linked QTL reported previously [2] but appears to be very closely located with seed dormancy linked QTL on chromosome 5HC in a population generated from Stirling and Harrington barley varieties [19]. The chromosome 5H QTL may be the same locus associated with seed dormancy in these studies. Salinity stress tolerance QTL at germination stage was mapped on chromosomes 4H, 5H and 6H in barley Steptoe/ Morex DH population; and on chromosomes 1H and 5H in Harrington/ TR306 doubled haploid population of barley [8]. These QTL are located on different chromosomes to the ones identified in our study.

Seedling growth stages salinity stress tolerance assessed in our study are controlled by nine QTL located on chromosomes 2H, 3H, 4H and 6H (Fig 3, Table 3)., A QTL on chromosome 2H identified by Bmag0125 marker and a QTL on chromosome 3H identified by marker bPb-6504 or bPb-1609 are linked with fresh weight per plant and dry weight per plant. The QTL on chromosome 2H is located at 80 cM distance and contributed by salinity stress sensitive Australian barley variety Gairdner. This QTL was linked with three traits namely fresh weight per plant and dry weight per plant in salinity stress treatment induced at first leaf full expansion growth stage, and fresh weight per plant recorded in control treatment. The QTL on chromosome 2H appears to be located farther apart from a QTL reported previously [2] at 45–50 cM distance linked with dry weight per plant at late growth stage in salinity stress condition in the CM72 x Gairdner DH population. This may suggest that different genetic mechanisms control salinity stress tolerance at seedling and late growth stages. When similar growth stages but different growth environments are considered, a study conducted on Yangsimai 1 x Gairdner DH population revealed that salinity stress tolerance linked QTL were closely located by 8 cM on chromosome 2H in a waterlogged and drained conditions [20]. Salinity stress tolerance linked QTL identified at 80.0 cM position in our study in the CM72 x Gairdner DH population is located distantly from the QTL that controlled salinity stress tolerance and developmental stage identified in the Yangsimai 1 x Gairdner DH population [20]. In a study that assessed salinity tolerance of a DH population derived from Yuyaoxiangtian (tolerant parent) and Franklin (susceptible parent), 5 salinity tolerance linked QTL accounting for more than 50% phenotypic variation were mapped on chromosomes 1H, 2H, 5H, 6H and 7H [21]. The QTL reported by [21] located on chromosome 2H and 6H were located at a distance of 32 cM and 36.6 cM respectively from stress tolerance linked QTL identified in our study. This indicates that genomic regions linked with salinity tolerance in the CM72 x Gairdner DH population of the current study is different from those identified in the Yuyaoxiangtian and Franklin DH population.

The article "Early growth stages salinity stress tolerance in CM72 x Gairdner doubled haploid barley population" was published in 2017. Journal: PLoS One.

The CM72 contributed QTL mapped on chromosome 3H at a distance of 176.5 cM is linked with three traits. These traits are fresh weight per plant in salinity stress induced at first leaf full expansion growth stage, dry weight per plant in salinity stress induced at seedling emergence and first leaf full expansion growth stages. This multi-traits controlling QTL on chromosome 3H identified in our study is mapped at the same location as spikes per line controlling QTL but located slightly distantly from a QTL linked with dry weight per plant at late growth stage in salinity stress free condition [2]. Dry weight per plant linked QTL at late growth stage reported previously [2] is located in a close proximity to the QTL mapped on chromosome 3H at 192.8 cM distance linked with fresh weight per plant in salinity stress treatment induced at seedling emergence. [22] studied CM72 x Gairdner DH population for salinity stress tolerance and identified grain yield linked QTL on chromosome 3H at 58.9 cM distance in salinity stress treatment, which was distantly located from biomass linked QTL on chromosome 3H in control as well as varying level of salinity stress treatment of our study. Shoot dry weight and leaf injury score linked QTL were rather mapped on chromosome 1H in 296 barley accessions originated from Asia [23].

When genetic factors linked with germination stage salinity stress tolerance are compared with those at seedling growth stages, our study revealed that QTL linked with salinity stress tolerance at these two different growth stages are located at a distance of 76.6–80.2 cM apart on chromosome 2H of the CM72 x Gairdner DH population. Germination stage salinity tolerance on chromosome 5H is not linked with any other traits assed in our study. Result from this study partly substantiates previous reports [8] that demonstrated that salinity stress tolerance conferring QTL at germination stage were different from those QTL linked with seedling growth stages salinity tolerance. Salinity tolerance QTL at germination in the DH lines of Steptoe/Morex were located on chromosomes 4H, 6H, and 5H, and in the DH lines of Harrington/TR306 on chromosomes 1H and 5H, while seedling growth stage stress tolerance were mapped on chromosomes 1H, 2H, 5H and 6H in Steptoe/ Morex DH population, and on chromosome 5H in Harrington/ TR306 doubled haploid population [8].

When association between genomic regions linked with plant height and those linked with biomass yield are compared, plant height linked QTL on chromosome 2H is located between QTL linked with germination stage tolerance at 41.6–48 cM distance and biomass yield linked QTL at 38.6 cM distance. This indicates that these QTL are independent genetic factors. However, QTL identified on chromosome 3H at 192.8 cM distance linked with fresh weight per plant in seedling emergence stage salinity stress and at 176.5 cM distance linked with biomass yield in seedling emergence and leaf expansion stages salinity stress is located at different chromosomal region from region linked with *sd1/ denso* gene in the Baudin x Ac Metcalfe barley DH population at about 55 cM distance [24]. The QTL in the Baudin x Ac Metcalfe DH population is in a very close chromosomal region to two QTL linked with plant height at maturity reported previously in the CM72 x Gairdner DH population in salinity stressed and non-stressed conditions [2]. A semi-dwarf 1 (*sdw1*) gene on chromosome 3HL control plant height in barley and sequencing of its different alleles locus points to HvGA20ox2 as the functional gene responsible for the phenotype [24, 25]. Plant height linked QTL in control and salinity stress environments were mapped at the same point on chromosome 3H and in close proximity on chromosome 5H in the TX9425 x Naso Nijo DH population [26]. The QTL on chromosome 3H reported by [26] is located at a different genomic regions to the QTL linked with plant identified in our study. Plant height linked QTL on chromosome 3H reported previously [2, 24] are distantly located from a QTL with the same function or seedling stage biomass yield identified in the current study. However, a QTL identified on chromosome 5H linked with germination percentage in 300 mM NaCl treatment of our study appeared to be located in a close proximity to plant height linked QTL in the TX9425 x Naso Nijo DH population [26].

The article "Early growth stages salinity stress tolerance in CM72 x Gairdner doubled haploid barley population" was published in 2017. Journal: PLoS One.

Adaptation to salinity stress in plants is often linked with three mechanisms, namely accumulation or synthesis of compatible solutes, antioxidant protection and regulation of ion homeostasis particularly Na+ and K+ homeostasis; the latter being acknowledged to play important roles in barley salinity tolerance [27]. Results from a study conducted on 189 Tibetan wild barley accessions showed that HvHKT1 gene is significantly associated with root Na+ concentration under saline environment and up-regulated immediately after salt stress, while HvHKT2 is substantially down-regulated after salt stress corresponding to decreased K+ concentration in both shoots and roots of barley under salinity condition [27]. Na+ concentration controlling QTL on chromosome 2H [2, 20] and Na+:K+ ratio controlling QTL on 6H [2], on chromosome 1H and 5H [20] have been reported in the CM72 and Gairdner DH population [2] and Yangsimai 1 x Gairdner DH population [20]. The QTL on chromosome 2H reported by [2] was in a very close proximity to QTL linked with germination stage salinity stress tolerance but located distantly from QTL linked with biomass yield at seedling stage identified in our study. No QTL linked with K+ accumulation was identified in a study conducted on F1-derived DH population from Barque-73 (*Hordeum vulgare* ssp. *Vulgare)*, a selection from barley variety Barque and moderate Na+ excluder, and a wild accession CPI-71284-48 (*H*. *vulgare* ssp. *Spontaneum*) capable of limiting Na+ accumulation in the shoots [28]. Rather they reported a single strong Na+ accumulation linked QTL on chromosome 7H genetic map at 13.9 cM. This QTL did not correspond to the location of Na+ exclusion Nax1 and Nax2 and thus named as barley locus HvNax3. HvNax3 locus reduced shoot Na+ accumulation by 10–25% in plants grown in 150 mM NaCl [28].

The article "Early growth stages salinity stress tolerance in CM72 x Gairdner doubled haploid barley population" was published in 2017. Journal: PLoS One.

Response to environmental stress such as salinity stress not only affect germination, biomass yield, grain yield, physiological traits but also phenology traits [2, 4–9, 20, 21, 28, 29]. Late flowering DH lines of Yangsimai 1 x Gairdner showed greater tolerance than early flowering lines with QTL associated with plant development genes showing significant effects on salinity tolerance in summer trials [20]. Although QTL associated with flowering time on chromosome 2H and 5H were reported to be overlapped with those for salinity tolerance in the Yangsimai 1 x Gairdner DH population [20], these QTL appeared to be located at different chromosomal regions to QTL identified in our study. This corroborates an observation made from a consensus QTL map reported by [29] that reflected phenology controlling genes reported from elsewhere and seedling stage biomass yield linked QTL identified in this study are located distantly. In general, it can be concluded salinity stress tolerance linked genes at germination stage, seedling growth stages, plant height and phenology genes are likely controlled by independent genetic factors.

### Application for marker assisted selection

Salinity stress tolerant parental genotype CM72 yielded higher fresh weight per plant and dry weight per plant than salinity sensitive Australian barley variety Gairdner in salinity stress treatment induced at first leaf full expansion growth stage. The fact that there is very highly significant Spearman’s genotypic rank correlation coefficient (r = 0.98^**^) between fresh weight per plant and dry weight per plant in individual treatments (Table 2), these two traits and QTL linked with them can be used as important genetic tools to select for salinity stress tolerance in early growth stages of barley. Particularly, the CM72 contributed QTL located on chromosome 3H is associated with fresh weight per plant and dry weight per plant in salinity stress induced at seedling emergence or first leaf full expansion growth stage is an important genetic tool in selecting for salinity stress tolerance at early growth stage.

## Concluding remarks

Salinity impairs barley germination and biomass yield at seedling growth stages. High phenotypic and genetic variation exists in the CM72 x Gairdner barley doubled haploid population. QTL linked with salinity stress tolerance at germination are different from those QTL linked with salinity tolerance at seedling growth stages. Particularly salinity stress tolerant CM72 contributed QTL on chromosome 3H linked with bPb-6504 marker linked with biomass yield in salinity stress treatments is an important genomic region that can be used for marker assisted selection in improving barley varieties for production in environments prone to salinity stress.

The article "Early growth stages salinity stress tolerance in CM72 x Gairdner doubled haploid barley population" was published in 2017. Journal: PLoS One.

## Abbreviations

DH: Doubled Haploid
QTL: Quantitative Traits Loci/ Locus
NST: Nutrient Solution Tank
RST: River Sand Tank
